The article "Agomelatine Softens Depressive-Like Behavior through the Regulation of Autophagy and Apoptosis" was retracted in 2024. Reasons: suspected computer-generated content; unreliable results or conclusions; concerns about the data; concerns about the results or conclusions.

# Agomelatine Softens Depressive-Like Behavior through the Regulation of Autophagy and Apoptosis

**DOI:** 10.1155/2021/6664591

**Published:** 2021-03-17

**Authors:** Fengpei Chen, Shijia Chen, Jie Liu, Nashwa Amin, Weidong Jin, Marong Fang

**Affiliations:** ^1^The Second Clinical Medical College of Zhejiang Chinese Medical University, Hangzhou 310053, China; ^2^Institute of Neuroscience, Zhejiang University School of Medicine, Hangzhou 310058, China; ^3^Department of Zoology, Faculty of Science, Aswan University, Egypt; ^4^Zhejiang Mental Health Center, Tongde Hospital of Zhejiang province, Hangzhou 310012, China

## Abstract

Depression is a common and disabling mental disorder with high recurrence rate. Searching for more effective treatments for depression is a long-standing primary objective in neuroscience. Agomelatine (AGO) was reported as an antidepressant with unique pharmacological effects. However, its effects and the underlying mechanism are still unclear. In this study, we sought to evaluate the antidepressant effects of AGO on the chronic restraint stress (CRS) mouse model and preliminarily investigate its effects on the gut microbial metabolites. The CRS model mice were established in 28 days with AGO (60 mg/kg/day, by oral) or fluoxetine (15 mg/kg/day, by oral) administration. The number of behavioral tests was conducted to evaluate the effect of AGO on depression-like behavior alleviation. Meanwhile, the expression of the BDNF/TrkB/pERK signaling pathway, apoptosis, autophagy, and inflammatory protein markers were assessed using western blot and immunofluorescence. Our findings show that AGO can attenuate the depressive-like behavior that significantly appeared in both sucrose preference and forced swimming tests. Additionally, a noticeable upregulation of autophagy including Beclin1 and LC3II, microglial activity marker Iba-1, and BDNF/TrkB/pERK signaling pathways are indicated. An obvious decreased expression of NF-*κ*B, iNOS, and nNOS as well as apoptosis including Bax is observed in AGO administration mice. On the other hand, we found that AGO impacted the rebalancing of short-chain fatty acids (SCFAs) in mouse feces. Altogether, these findings suggest that AGO can exert antidepressant effects in a different molecular mechanism.

## 1. Introduction

Depression is characterized by sadness, anhedonia, low self-esteem, loss of motivation, sleep disruption, loss of appetite, and other cognitive symptoms [1]. Symptoms of depression are highly prevalent, affecting up to 27% of the general population according to recent meta-analytic data [2]. However, the exact biological, psychological, and social mechanisms underlying the pathogenesis of depression remain largely unknown. Currently, most patients with depression are treated with synthetic drugs including selective serotonin reuptake inhibitors (SSRI) that act on the monoaminergic system, serotonin-norepinephrine reuptake inhibitors (SNRIs), tricyclic antidepressants (TCAs), norepinephrine and dopamine reuptake blockers, and monoamine oxidase inhibitors which exhibit little or no improvement on depression and have side effects such as fatigue, sleep disorders, cognitive disorders, and sexual dysfunctions [3–5].

AGO is an antidepressant with unique pharmacological actions. Previous studies reported AGO to act as both a melatonin agonist and a selective serotonin antagonist [6]. In the previous decade, AGO was reported to have at least comparable efficacy to other antidepressants in terms of response and remission rates and to confer better tolerability and be associated with fewer side effects [7–9]. In vertebrates, the pineal gland is the main source of melatonin production. Of the many substances identified, recent studies suggest that melatonin and its metabolites are highly effective physiological antioxidants and can also exert direct, non-receptor-mediated actions, such as the scavenging of a number of free radicals including both reactive oxygen and nitrogen species (ROS and RNS, respectively) [10–13].

BDNF is associated with neuropsychiatric disorders, such as depression [14] and schizophrenia [15]. BDNF and its mechanisms are also therapeutic targets of pharmacological agents that are currently used to treat mice with depression [16]. Previous studies have shown that fluoxetine can improve depression-like behaviors by regulating the BDNF signaling pathway [17]. However, the role of BDNF in the antidepressant process of AGO still requires in-depth research. Ample preclinical evidence suggested that exposure to acute or chronic stress agents triggers the production of cytokines, which may be related to the physiological processes mediated by autophagy [18]. The induction of autophagy protects neurons and glial cells under stress through the deregulation of various DAMPs and suppression of stress reaction, which will contribute to the alleviation of depression [18, 19]. The observation that the increase in autophagic markers goes along with the reversal of the behavioral effects argues in favor of autophagy being a beneficial component of the stress response in general [20]. Existing research shows that fluoxetine could promote the autophagic flux unblocked in the way of enhancing fusion of autophagosomes with lysosomes in primary astrocytes and finally ameliorates depression [21]. Similarly, apoptosis, another molecular mechanism that maintains cellular homeostasis, has recently been shown to be closely related to the development of depression [22]. Moreover, autophagy is important in cell death decisions and can protect cells by preventing them from undergoing apoptosis [23]. All of these indicate that autophagy and apoptosis may act as key mediators in antidepressant and stress-induced behavioral action.

However, whether AGO can alleviate depression by regulating autophagy or apoptosis is currently not clearly understood. In the current study, we aimed to investigate (i) the underlying mechanisms of AGO administration in CRS-induced depression, (ii) the changes in the hippocampus and subsequent anxiety behavior, and (iii) the impact of the AGO regimen on brain inflammation factors and microbial metabolites such as SCFAs.

## 2. Materials and Methods

### 2.1. Animals

Male C57BL/6N mice (weighing 20 ± 2 g, 8 weeks old) were used in this study. The mice were maintained in a room at 24 ± 1°C with 50%–60% relative humidity under a 12 h light/dark cycle (lights on at 09:00) with free access to food and water. All experimental procedures were approved and performed according to the Animal Care and Use Committee of the Institute of Zhejiang University, China. The animal ethics number is ZJU20160267.

### 2.2. Study Design and Drug Administration

After 2 weeks of adaptation, the mice were randomly assigned to 4 groups of 8 mice each: control (CON), chronic restraint stress (CRS), fluoxetine (FLX), and agomelatine (AGO). All groups were subjected to CRS except the control group. Fluoxetine (Patheon, France) and agomelatine (Lianyungang, China) were dissolved in physiological saline (NaCl, 0.9%). Dose and administration schedules of AGO and FLX were based on previous results [24]. Specifically, mice in the CRS group were subjected to CRS and intragastric administration of 8.0 mL/kg saline daily, and AGO and FLX were administered to mice at doses of 60 mg/kg body weight/day and 15 mg/kg body weight/day, respectively. Drugs were administered half an hour before the CRS regimen. The specific experimental procedure is shown in Scheme 1.

### 2.3. The Chronic Restraint Stress Model

The CRS model was based on the Chiba method [25], with slight modification. Briefly, mice were individually restricted in a modified, well-ventilated tube for 6 h without water and food, and mice were exposed to CRS for 28 consecutive days.

### 2.4. Behavioral Test

#### 2.4.1. Open Field Test (OFT)

The apparatus consisted of a white Plexiglas box (45 cm × 45 cm × 45 cm) divided into two zones: outer square (periphery) and inner square (center: 25 cm × 25 cm). Each mouse was placed in the center of the box and allowed to freely explore the environment in a room with dim light for 5 min. The movement of the mouse was recorded by a video camera (VideoTrack, Viewpoint Inc., France). The total distance covered in the box and the time spent in the central zone were calculated.

#### 2.4.2. Elevated Plus Maze (EPM)

The elevated plus maze apparatus consisted of two opposite-facing closed arms (30 cm × 5 cm × 15 cm), two opposite-facing open arms (30 cm × 5 cm), and a central area (5 cm × 5 cm), and the maze was 50 cm above the ground. For the elevated plus maze, the mouse was placed in the center of the maze facing one of the two closed arms. A 5-minute test was recorded using an automatic analyzing system (ANY-maze, Stoelting, USA). The number of entries and the time spent in the open arms were recorded using an automatic analyzing system.

#### 2.4.3. Forced Swimming Test (FST)

Mice were placed into a cylinder (12 cm diameter, 25 cm height) filled with 24 ± 1°C water. Water depth was adjusted so that the mice can neither touch the bottom nor jump out. Two mice at a time were videotaped from the side. A cardboard divider separated the cylinders so that the mice could not see each other during the trials. The mouse activity was video recorded for 6 min, and the duration of immobility was recorded during the last 4 min of the 6 min test. After the test session, mice were placed in a clean cage containing paper towels under a heat lamp until dry. Immobility was defined according to criteria described [26].

#### 2.4.4. Sucrose Preference Test (SPT)

The SPT was performed as previously reported [17] with slight modification. Briefly, mice were single housed and were accustomed to two bottles of water after two bottles of 2% sucrose for a day. After being deprived of water and food for 24 h, the mice were exposed to one bottle of 2% sucrose and one bottle of water for 2 h during the dark phase. Bottle positions were switched after 1 h (for a 2 h test). After 2 hours of testing, water and sucrose consumption was measured.

### 2.5. Western Blot

Mice were sacrificed by cervical dislocation. The hippocampus was extracted for the evaluation of protein level and stored at -80°C until use. Total protein of the hippocampus was prepared from each group using 1 mL ice-cold RIPA buffer, supplemented with 1% PMSF (phenylmethanesulfonyl fluoride, Beyotime ST505), protease inhibitors, and phosphatase inhibitors. Probes were ground and then centrifuged at 12,000 rpm for 30 min at 4°C before protein supernatants were obtained. The protein concentration was determined by using the BCA assay. 20 *μ*g protein was electrophoresed on a 10% SDS-PAGE gel and transferred onto a polyvinylidene difluoride (PVDF) membrane. After blocking with 5% nonfat milk in TBS-Tween 20, membranes were incubated with primary antibodies overnight at 4°C as follows: rabbit anti-NF-*κ*B/p65 (Cell Signaling Technology, 1 : 1,000), rabbit anti-nNOS (Omnimabs, 1 : 500), rabbit anti-iNOS (Boster, 1 : 500), rabbit anti-LC3B (Novus, 1 : 1000), rabbit anti-p62 (Cell Signaling Technology, 1 : 1000), rabbit anti-Beclin (Cell Signaling Technology, 1 : 1000), rabbit anti-Bax (Boster, 1 : 500), rabbit anti-Bcl2 (ABclonal, 1 : 500), rabbit anti-BDNF (Boster, 1 : 500), rabbit anti-TrkB (Abcam, 1 : 1000), rabbit anti-pERK (Cell Signaling Technology, 1 : 1000), and mouse anti-GAPDH (ABclonal, 1 : 10000). Then, the membranes were subjected to three washing steps with TBS-Tween 20 (each 5 minutes) before incubation with the secondary antibody goat anti-rabbit IgG antibody (Bioker, 1 : 5000) and goat anti-mouse IgG antibody (Bioker, 1 : 5000) at room temperature for 2 h. After the final washing steps, membranes were subjected to enhanced chemiluminescence reaction and bands were quantified by densitometry (Quantity One 4.2, Bio-Rad, Hercules, CA). Densitometric values of markers were normalized to GAPDH levels. Each experiment was performed at least three times. The detection and quantification of each band were performed using Image Lab software.

### 2.6. Immunofluorescent Staining

Mice were perfused with 4% paraformaldehyde (PFA) after being perfused through the heart with 50 mL (±) of saline. Brain tissue sections were subjected to immunohistochemistry analysis. Frozen sections, about 16 *μ*m thick, were rinsed in 0.01 M PBS for 5 min and then moved to room temperature for 1 h and blocked with 5% normal goat serum. Incubation with primary antibodies occurred overnight at 4°C: Iba1 (Abcam, 1 : 100). The sections were washed with 0.01 M PBST for 5 min three times on the following day and then incubated with secondary antibodies containing FITC goat anti-rabbit IgG (1 : 100, Boster, BA1105) and Alexa Fluor® anti-rabbit 488 for 3 h in the dark at room temperature. After washing, probes were mounted in medium containing DAPI (VECTASHIELD, USA). A fluorescence microscope (Olympus BX61, NIKON, Japan) was used for taking images. IBa1 staining was obtained with the NIH ImageJ software (https://imagej.net/welcome).

### 2.7. Fecal SCFA Detection: Gas Chromatographic Analysis

The fecal samples were frozen immediately after collection and stored -80°C until analysis. Specifically, 80 mg of each fresh stool sample was weighed, suspended in 500 *μ*L anhydrous alcohol, and homogenized for approximately 5 min. Then, the sample was incubated at room temperature for 10 min with occasional shaking and centrifuged for 10 min at 12,000 rpm. The supernatant was transferred into 2 mL screw top vials (Agilent, United States). The concentration of SCFAs (including acetate, propionate, butyrate, isobutyrate, and valeric acid) in mouse fecal samples was determined using an Agilent 7890A gas chromatography unit, fitted with a high-resolution gas chromatography DB-624 column (30 m × 0.32 mm × 1.8 *μ*m, Agilent, United States). Nitrogen was supplied as a carrier gas at a flow rate of 1.2 mL/min. The initial oven temperature was 100°C, maintained for 5.0 min, raised to 200°C at 20°C/min, and finally held at 200°C for 5 min.

### 2.8. Statistical Analysis

Normalization and equal variances between group samples were assessed using the normal *Q*-*Q* plot and homogeneity test for variance, respectively. When normalization and equal variance between sample groups were achieved, one-way ANOVA with LSD was used. Where normalization or equal variance of samples failed, Mann–Whitney *U* tests were performed. Each value was presented as a mean ± SEM and analyzed with one-way ANOVA using SPSS 22.0 software. A value of *P* < 0.05 was considered significant.

## 3. Results

### 3.1. AGO Ameliorates CRS-Induced Depressive-Like Behavior

In order to investigate the effect of AGO in the depressive-like behavior, we sought to first analyze the body weight during CRS and drug treatment. No significant differences were found in the baseline body weight among the four groups. Then, statistical analysis revealed that CRS resulted in retardation of the body weight gain starting with day 9 compared to the control group, while AGO and FLX treatment did not counteract the effect (Figure 1(a)). At the end of the chronic stress period, a battery of well-established behavioral tests aimed at measuring anxiety-like behavior (OFT, EPM) and depression-like behaviors (SPT, FST) were conducted. Mice in the CRS group showed significant longer freezing time in FST (Figure 1(b)) and lower sucrose preference (Figure 1(c)) compared with the control mice. AGO and FLX significantly restored the above changes. Unfortunately, no significant effect was observed in the locomotor activity and the time spent in the central area (Figures 1(d) and 1(e)). In addition, the CRS procedure did not alter entries into and time spent in the open arms (Figures 1(f) and 1(g)). These experiments suggest that AGO restores the depressive-like behavior after CRS.

### 3.2. Effect of AGO Treatment on BDNF/TrkB and ERK1/2 Activity

Recent studies demonstrate that BDNF-TrkB signaling is required for promoting proliferation [27] of newborn neurons in the adult hippocampus in response to antidepressant administration. Previous studies were conducted in order to determine if AGO administration alters the level of BDNF in the hippocampus [14], a region implicated in the actions of antidepressants. Indeed, expression of BDNF and TrkB declined in the hippocampus of mice subjected to CRS as depicted in Figures 2(a)–2(c). This was corroborated with decreased levels of active ERK1/2 (Figures 2(a) and 2(d)). Interestingly, AGO restored the CRS-induced decrease to levels achieved by FLX regimens. Moreover, there was no significant change between the AGO and FLX groups, indicating that these two drugs protect similarly against CRS-induced depressive symptoms by interfering with BDNF and TrkB expression and ERK activity in the hippocampus.

### 3.3. AGO Promotes CRS-Induced Autophagy in the Hippocampus

To confirm the protective effect of AGO on hippocampal autophagy in the CRS model, we sought to investigate the putative protective mechanisms of AGO. Therefore, the expression level of autophagy markers LC3II, p62, and Beclin1 was analyzed by western blotting. Our experiments showed that Beclin1 was downregulated in the CRS group (Figures 2(e) and 2(f)), which was restored in AGO-treated mice comparable to the levels found in animals subjected to FLX regimens. Similarly, LC3 II expression in the hippocampus increased in mice subjected to AGO and FLX treatment after CRS (Figures 2(e) and 2(g)). Given that LC3II and Becline1 can only reflect the initialization of autophagy, we also detected the protein level of p62, which is the best-characterized molecule and degradation product of autophagy. As shown in Figures 2(e) and 2(h), hippocampal p62 levels were increased in CRS mice but significantly decreased after treatment with AGO and FLX. The results suggest that stress led to lower levels of autophagy after the chronic restraint stress; this was ameliorated by AGO treatment having higher levels than stressed animal.

### 3.4. AGO Decreases CRS-Induced Apoptosis in the Hippocampus

To confirm the role of AGO treatment in the apoptosis mechanism, we investigated the hippocampal Bax and Bcl-2 protein levels to evaluate apoptosis. As shown in Figures 2(i) and 2(j), CRS resulted in a decrease in the Bcl2/Bax ratio in the hippocampus. Administration of AGO was associated with a significantly increased Bcl2/Bax ratio in the hippocampus. Altogether, these findings suggest that AGO might improve depressive symptoms in the CRS mouse model by maintaining essential autophagy and inhibiting excessive apoptosis.

### 3.5. AGO Treatment Alleviates CRS-Induced Inflammation in the Hippocampus

Ample preclinical and clinical evidence showed that external stress is accompanied by an increased production of proinflammatory cytokines and their upstream regulators. NF-*κ*B is a transcription factor reported to regulate a plethora of proinflammatory cytokines, such as iNOS [28]. Our experiments show that NF-*κ*B subunit p65/RelA is elevated after CRS in the hippocampus (Figures 2(k) and 2(l)). Furthermore, our data show that iNOS and nNOS are also elevated after CRS (Figures 2(k), 2(m), and 2(n)). Most importantly, administration of AGO partially restored both p65 and iNOS/nNOS levels, which were comparable with FLX treatment (Figures 2(k), 2(m), and 2(n)). Altogether, these findings implicate NF-*κ*B in CRS-induced inflammation.

### 3.6. Effect of AGO Treatment on Alterations of Microglia in the Mouse Hippocampus

To investigate the effect of AGO and FLX on microglia in the hippocampus, immunofluorescence staining for hippocampal sections was performed. IBa1 was used as a specific marker for microglia. CRS administration resulted in a decrease in IBa1 expression in the hippocampal region (Figures 3(a) and 3(b)). Importantly, AGO treatment ameliorated IBa1 expression compared with that of CRS mice (Figures 3(a) and 3(b)) in line with data presented in Figure 2.

### 3.7. Changes in SCFA Concentrations

Based on the “microbiota-gut-brain” axis, we determined the effects of AGO administration on short-chain fatty acids. The SCFA (acetate, propionate, isobutyrate, butyrate, and valeric acid) concentration in mouse fecal samples was analyzed by GC and is shown in Figure 4. Of all investigated fatty acids, only isobutyrate showed a difference between CRS and control. Administration of AGO mainly decreased the concentration of acetate, valeric acid, and total SCFAs and not isobutyrate. On the other hand, high levels of isobutyric acid induced by CRS were relieved by drug treatment indicating that established AGO or FLX regimens can attenuate depressive-like behaviors via the modulation of microbiota-driven SCFA levels.

## 4. Discussion

In our present study, we found that AGO treatment for 4 weeks alleviated depression-like behaviors via activating autophagy and the BDNF-TrkB pathway in the hippocampus of CRS mice. Moreover, an obvious decrease in inflammation including NF-*κ*B, iNOS, and nNOS as well as apoptosis including Bax is confirmed. It implies the possibility that regulating autophagy and the BDNF-TrkB pathway may be an alternative mode of action for AGO besides its role in modulating melatonin.

CRS is a noninvasive protocol, which is very similar to human psychological stress [29] and therefore renders as a reliable animal model of studying the depression with good replicability. Our findings revealing lower body weight gain and depressive-like behaviors (FST and SPT) after CRS are consistent with previous studies [30]. Contradicting literature reported either the failure of CRS to generate an anxiety-like behavior or an important role of CRS in inflicting such behavioral changes [31–33]. Reasons for this discrepancy might be attributed to the parameters of the applied restraint stress (e.g., frequency and duration) [34]. In short, the successful establishment of depression model mice allowed us to study the antidepressant mechanism of AGO.

BDNF-related signaling pathways have been reported to play an essential role in the pathogenesis of stress-induced depression-like behaviors [35]. In the present study, we found that expression levels of BDNF/TrkB in the hippocampus of the CRS group were significantly downregulated. This is consistent with the current clinical research results [36]. Such BDNF/TrkB [37] integration leads to the activation of some signaling pathways including extracellular signal-regulated kinase 1/2 (ERK1/2) which is consistent with our findings that CRS-induced depressive-like behaviors and the consequent downregulation of BDNF/TrkB and ERK1/2 activity could be reversed by AGO administration.

In fact, autophagy and apoptosis constitute a strategy to adapt to and cope with the stress. The two affect each other and form a complex molecular regulatory network [38]. Stress is known to predispose rodents to depressive-like behaviors via inducing apoptosis in the hippocampus of mice [39]. Studies have shown that knocking out the proapoptotic factor Bax can reduce anxiety and depression-like behaviors in a mouse model of stress [40]. Analogously, enhanced apoptosis was detected in the hippocampus of rats tested in a repeated unpredictable stress model of depression [22]. The results of the present study indicate that AGO acts as an antidepressant partly through its role in improving the ratio of Bcl2/Bax. In many cases, autophagy usually manifests well before apoptosis “dismantles” the cell. Preclinical experiments have found that signs of decreased autophagy appeared in both chronic unpredictable stress and LPS-related depression model [41, 42]. Our results confirmed that CRS does cause differences in the expression of autophagy and apoptotic factors in the hippocampus; i.e., CRS results in increased p62 and decreased Beclin1. Unfortunately, we did not find any differences upon LC3II expression. However, the features of depression could be prevented through increased autophagy and antiapoptosis activity as a result of AGO or FLX administration. This is consistent with our previous research on the antidepressant mechanism of FLX [43]. Therefore, we think that this might represent a potential antidepressant mechanism orchestrated by AGO.

SCFAs are the key molecules that modulate microglial maturation and function, as well as depression [44–46]. In other studies, the mechanism of melatonin receptor expression may involve the action of SCFAs [47], and this effect does not necessarily affect the signals of brain neurons. It may be manifested by altering brain inflammation, affecting neuronal BDNF or autophagy pathways. Results from this study indicate that the CRS procedure can significantly increase isobutyrate level in feces and decrease IBa1 expression in the hippocampus indicating that isobutyrate plays an important role in the CRS procedure and may be involved in regulating the expression of IBa1. As microglia are the resident immune cells in the brain, they normally respond to various neuropathological stimuli, including stress, injury, and infection [48]. Once activated, a rapid proliferation in microglial densities and morphological changes result, followed by the release of proinflammatory and anti-inflammatory cytokines [49]. In this study, we found that CRS-induced depression is accompanied by elevated proinflammatory cytokine regulators such as transcription factor NF-*κ*B or increased iNOS, in line with previous studies [50]. As a novel antidepressant, AGO can rebalance the above changes to exert an antidepressant effect. In other words, AGO can exert antidepressant effects through immune pathways. More importantly, for the changes in the content of isobutyric acid induced by CRS, we found that AGO could not reverse the disordered concentration but FLX did. The possible reasons might be related to the different molecular mechanisms of the two drugs.

## 5. Conclusion

Taken together, these data provide further evidence for a beneficial role of AGO and its effects in the hippocampus under stressful conditions and confirmed that AGO can protect the CRS mice from depression. AGO may funnel its antidepressant effect through part of the molecular pathways delineated in the above, further confirming the important role of these cellular events in depression, and therefore might be used as an antidepressive drug in CRS.

## Figures and Tables

**Scheme 1:** Experimental schedule. Mice were treated for a total of 4 weeks with agomelatine, fluoxetine, or saline. After 4 weeks of treatment, animals underwent a battery of tests relevant to depression. All groups were sacrificed on the same day. Tissues were harvested for further analysis. CRS: chronic restraint stress; OFT: open field test; FST: forced swimming test; SPT: sucrose preference test.

**Figure 1:** CRS-induced depression-like behaviors in mice. (a) Effects of CRS and drug treatment on body weight are presented. (b) The immobility time in FST after CRS, AGO, and FLX treatment is shown. (c) SPT after CRS and drug treatment is depicted. (d) Total distance traveled in the OFT after CRS and drug treatment is presented. (e) Time spent in the center area in OFT after CRS and drug treatment is presented. (f) Open arms entry in the EPM is shown. (g) Time in open arms in the EPM after CRS and drug treatment is shown. ^∗^*P* < 0.05; ^∗∗^*P* < 0.01; ^∗∗∗^*P* < 0.001; ns = not significant. The values represent mean ± SEM. *n* = 8.

**Figure 2:** Effect of AGO treatment on BDNF/TrkB and pERK1/2 in autophagy, apoptosis, and inflammation in CRS mice. (a) Representative western blot results of BDNF, TrkB, and pERK1/2 are shown; densitometry analysis of BDNF (b), TrkB (c), and pERK1/2 (d) in the hippocampus is presented. (e) Representative western blot results of LC3II, Beclin1, and p62 are shown; densitometry analysis of Beclin1 (f), LC3II (g), and p62 (h) in the hippocampus. (i) Representative western blot results of Bcl2 and Bax are shown; (j) densitometry analysis of the Bcl2/Bax ratio in the hippocampus. (k) Representative western blot results of NF-*κ*B/p65, iNOS, and nNOS; densitometry analysis of NF-*κ*B/p65 (l), iNOS (m), and nNOS (n) in the hippocampus. ^∗^*P* < 0.05; ^∗∗^*P* < 0.01; ^∗∗∗^*P* < 0.001; ns = not significant. The values represent mean ± SEM. *n* = 3-5.

**Figure 3:** Immunofluorescence results indicated variation of microglial activation after CRS and AGO treatment. (a) Representative images of Iba1 (green) and DAPI (blue). Merged images are shown in the right panel. Scale bar = 100 *μ*m. (b) Quantification analysis of Iba1-positive cells in the DG of the hippocampus. ^∗^*P* < 0.05; ^∗∗^*P* < 0.01; ns = not significant. Values are expressed as mean ± SEM. *n* = 3.

**Figure 4:** Effects of AGO on CRS-induced SCFA changes in fecal samples. ^∗^*P* < 0.05; ^∗∗^*P* < 0.01; ^∗∗∗^*P* < 0.001; ns = not significant. The values represent mean ± SEM. *n* = 8.

## Data Availability

The data used to support the findings of this study are available from the corresponding author upon request.
